# Internet of Things and Robotics in Transforming Current-Day Healthcare Services

**DOI:** 10.1155/2021/9999504

**Published:** 2021-05-26

**Authors:** Bikash Pradhan, Deepti Bharti, Sumit Chakravarty, Sirsendu S. Ray, Vera V. Voinova, Anton P. Bonartsev, Kunal Pal

**Affiliations:** ^1^Department of Biotechnology and Medical Engineering, National Institute of Technology, Rourkela 769008, India; ^2^Department of Electrical Engineering, Kennesaw State University, Marietta Campus, Marietta, GA 30060, USA; ^3^Faculty of Biology, M. V. Lomonosov Moscow State University, Moscow 119234, Russia

## Abstract

Technology has become an integral part of everyday lives. Recent years have witnessed advancement in technology with a wide range of applications in healthcare. However, the use of the Internet of Things (IoT) and robotics are yet to see substantial growth in terms of its acceptability in healthcare applications. The current study has discussed the role of the aforesaid technology in transforming healthcare services. The study also presented various functionalities of the ideal IoT-aided robotic systems and their importance in healthcare applications. Furthermore, the study focused on the application of the IoT and robotics in providing healthcare services such as rehabilitation, assistive surgery, elderly care, and prosthetics. Recent developments, current status, limitations, and challenges in the aforesaid area have been presented in detail. The study also discusses the role and applications of the aforementioned technology in managing the current pandemic of COVID-19. A comprehensive knowledge has been provided on the prospect of the functionality, application, challenges, and future scope of the IoT-aided robotic system in healthcare services. This will help the future researcher to make an inclusive idea on the use of the said technology in improving the healthcare services in the future.

## 1. Introduction

The advancements in modern technology have facilitated researchers and scientists in transforming healthcare services. The leading-edge technologies have been extensively applied in designing and implementing various medical devices that are used for diagnosis, treatment, monitoring, and testing. This has been possible not only due to the development of the clinical-grade sensors but also due to the sensor networks that are implemented in hospitals. The combination of the sensors and sensor network has significantly helped to optimize healthcare delivery from a remote location. Due to the aforesaid advancements, healthcare services have become more adaptable, accessible, and affordable. Some of the most widely used advanced technologies that are proficient in the revolution of healthcare applications include big data analytics, machine learning, artificial intelligence, cloud computing, computer vision, and the Internet of Things (IoT) [1–5]. Data analytics have shown potential in identifying patterns and hidden features from the health data and helps in improving the quality of healthcare through an efficient decision-making capability [6]. Moreover, artificial intelligence (AI) techniques including machine learning (artificial neural networks, deep learning, etc.) have also augmented the work of healthcare professionals by processing a huge amount of healthcare data that are available in the form of electronic health records. Some of the healthcare applications of AI include diagnosis of respiratory conditions using chest X-rays, early detection of cancers, heart diseases, and predicting human health conditions [7]. Similarly, in the case of surgeries and therapeutic applications, the various advanced imaging techniques, including computer visions and computer tomography, have been efficiently employed [5]. The use of cloud services in healthcare provides a platform to store, process, and share healthcare records and reports, patient's personal information, etc. This delivers more flexibility to the healthcare services by using intercloud infrastructures to share health information, generate bills, etc. [8]. Although numerous advanced technologies have recently emerged in the healthcare industry, the one that shows potential in employing multiple technologies into a single environment is the Internet of Things (IoT).

In recent years, IoT has shown great efficiency in meeting the healthcare needs of people. Internet of Things (IoT) represents a network that connects multiple physical things (devices) through Internet connectivity. This allows unambiguous data and information sharing among the connected users. The integration of IoT technology can transform a device into a smarter, effective, and efficient device. Furthermore, IoT technology shows competence to connect the device with the real world. This has led to a substantial increase in the application of IoT technology in various sectors including healthcare. Experts believe that the IoT market in healthcare will hit more than 117 billion in 2021 [9]. The main contributors to this growing market are the sedentary lifestyle, the increased population, and the gradual spike in healthcare issues. Moreover, these aforesaid factors have also burdened the healthcare industry with the increase in the number of patients and new diseases with every passing day. Hence, it is more challenging to find a futuristic solution that provides more efficient and cost-effective healthcare services. In this regard, IoT is uncovering various other technologies, including robotics for better diagnosis, treatment, monitoring, and patient management. The integration of IoT and robotics provides an ecosystem where humans, robots, and IoT-system work cooperatively. The system is mostly inspired by the cloud-robotic system [10]. Cloud-robotic relies on “cloud computing” to access a large amount of data and process that information to perform specific operations. Herein, all operations, including sensing, computing, and memory, are integrated into a single network robot. The inclusion of robotic technology is meant to achieve some extent of human-like automation with a reduction in human intervention. This integrated system employs machine learning algorithms to program and train machines that will be able to perform in the medical environment. The system receives the patient's health information from the robotic system, shares these data through a network among the health professionals, and acts either based on the received feedback or using an intelligent computation. In recent days, IoT and robotics have been extensively applied in solving various healthcare problems from assisting the doctors remotely during surgery to providing rehabilitation to the differently abled [11–13]. Moreover, it is reducing the burden of medical personnel by relieving them from a routine task and making the medical procedure safer and cheaper than before. The use of robots allows for achieving higher accuracy and reducing human error. Although there is a remarkable evolution in the application of these two widely used technologies, the literature lacks comprehensive knowledge on the application of the integrated system where IoT and robotics will work cooperatively.

On this note, the current review aims to provide extensive information regarding the application of robotics and IoT technology in healthcare. Furthermore, we have discussed some of the most widely used applications of the IoT-aided robotic system in healthcare that includes assistive surgery, telepresence, rehabilitation, prosthetics, sanitization, and prescription dispensation. This review may form a reference for future researchers in deciding their prospects in the aforesaid field by highlighting the existing issues and future challenges.

## 2. Definition, Architecture, and Basic Functionalities of IoT-Aided Robotic System

The IoT-aided robotic system can be defined as a wireless network that provides advanced robotic services by interconnecting multiple robots with the smart environment (Figure 1). It also makes use of advanced information and communication technologies such as cloud computing and big data analytics that enables the robotic system to share information and make use of the enormous amount of data stored in the cloud. Earlier studies in the field of robotics were mostly focused on increasing robot autonomy, perception, and data processing, which are important criteria for the independent functioning of a robot. However, in the IoT-aided robotic system, the functionalities of a robotic system are integrated with various sensors to achieve a common healthcare goal. Besides monitoring, diagnosing, and performing simple tasks, the integrated systems are designed to perform complex operations. Furthermore, at the same time, the sensor information from the smart environment can be efficiently shared and used by the robotic system. In simple words, the IoT-aided robotic system can be defined as an extension of the IoT that possesses the advantage of robotic technology.

The architecture of an IoT-aided robotic system consists of three layers: the physical layer, network control layer, and the application layer. Since the architecture of the integrated system is not the primary focus of this study, only a brief introduction to the architecture is provided herein. However, a detailed description of the architecture is given in [15]. The sensors are used for collecting the vital health information of the patient's body and information depicting the surrounding environment. This layer also includes switches, actuators, and other drives that can be used to perform simple actions. Robots are intelligent devices that can connect either with other robots to create a multi-robot network or with sensors/actuators. The network layer is responsible for all the interconnections within the network sensors and the robots. It includes routers, controllers, and communication and network protocols. For information storage, the system may use local as well as remote storage using cloud computing technology. With help of the physical and network layer, the application layer performs specific tasks using the information collected from the physical layer. The application layer architecture solely depends on the objective of the integrated system. However, depending on the healthcare applications and the nature of tasks, an IoT-aided robotic system must be able to show a set of functionalities to meet the demands. In this section, several such abilities (Figure 2) of an IoT-aided robotic system have been discussed in detail.

### 2.1. Perception Ability

Perception is defined as the ability of a system to perceive, understand, and sense the surrounding environment [16]. The perception ability of a robot makes the system efficient to perform complex tasks and allows it to function in diverse situations [17]. Furthermore, it enables a robotic system to access data from multiple sensors and record real-time information such as speech, image, and video. In the healthcare environment, the perception ability can be utilized to observe human behavior related to anomalous activities and unhealthy habits [18]. Presently, it has been used in various healthcare applications such as clinical measurements (blood pressure, temperature, and activity recognition), disease diagnosis, monitoring patient's recovery, and disinfecting/cleaning of hospital premises [19, 20]. Instead of placing a sensor onboard, the use of a mobile robot allows collecting of information from the flexible and dynamic positions. Furthermore, the sensing and data analytics technology that is used in IoT provides a wider perspective to robots as compared to local sensing. This lets the medical system implement time-resolved sensing strategies. One of the most challenging tasks during perception in an IoT-aided robotic environment is the ability to sense information that is distributed in space and time [21]. Hence, while designing an IoT-aided robotic system, it is of primary focus to use some techniques that allow the system to perceive the distributed information [22]. Moreover, the information regarding the location of a robot is also crucial as it helps in collecting environmental information. Despite, remarkable growth in this field, self-localization is continued to be a challenging task in more crowded areas and places where global positioning system (GPS) does not work properly. In that case, the integration of IoT provides reliable location information to domestic robots. This is achieved using various IoT-based communication technologies such as Radio-frequency identification (RFID), Wi-Fi, Zigbee, and Bluetooth [23].

### 2.2. Motion Ability

The motion ability can be an added value for a robotic system as it increases the working range of the system. Usually, in robotic systems, increasing of the working range is achieved with help of advanced mechanical design and using an efficient navigation system. The mechanical design helps in creating the movement while the navigation system helps in deciding the path for the motion. A perfect navigation system enhances the comfort of the patients during assistance. The use of IoT technology may help in assisting the robotic system to achieve some extent of human-like automation in various healthcare services. In addition, it collects information from different locations and acts collectively to perform specific operations such as lifting and moving patients and assisting patients to do their daily activities [24]. In some healthcare applications, a continuous movement of the robot is necessary as in the case of touring the caregiver's activity area or fall prevention. Herein, the robot has to find an optimal path to reach the destination efficiently by avoiding the obstacles in crowded areas. Hence, achieving efficient navigation is the prime focus in many researches. This is due to the inability of the traditional robot to handle a dynamic environment where there is a stochastic movement of people. Furthermore, due to the unpredictable movement of people, the avoidance of collision for a robotic system is difficult, particularly while working in a narrow space. Recently, numerous studies in the literature have addressed the issue of collision avoidance of robotic systems [25–27]. Safeea et al. in their study have proposed an online collision-avoidance system in a surgical environment. Herein, IoT is used to achieve this without any physical contact [28]. Mišeikis et al. have developed a healthcare robot called “Lio,” which is used for autonomously assisting staff and patients in a hospital. The robot uses a combination of visual, audio, ultrasound, laser, and a mechanical sensor for safe navigation that enables the robotic system to avoid collision [29]. In [30], a smart-walker called “Guido” has been proposed for visually impaired persons. The system uses a map-based navigation system that creates a map of its surrounding environment and also tracks its position. The system creates a path based on the generated map and uses a collision avoidance algorithm to reach a destination without any obstacle. When the healthcare environment is associated with multiple robots as in the case of surgery, it is important to have an alternate mode of communication among them. This is to avoid miscommunication among the robots after the loss of Internet connectivity.

### 2.3. Interaction Ability

The ability of an IoT-aided robotic system to interact with the users, operators, and various other systems that are present in the environment makes the system user-friendly and efficient. Moreover, it can act as a companion to the disabled and elderly people who need special attention [31]. Although the machine-to-machine interaction is well adopted in a robotic system, the integration of IoT technology can facilitate efficient human-robot interaction. The disadvantage of using the onboard sensors of the robotic system for detection is that it limits the range of operation. However, external sensors, cameras, and wearable sensors provide a broader perspective that enhances the interaction ability of a system. The physical expressions, voice, and gestures have been used not only for estimating the human emotional states but also to enable the robot to respond to these emotions. Various body-worn sensors have been used to predict human emotions. Chen et al. [32] have used human-robot interaction through hand gestures as a control mechanism for households and wheelchairs. Herein, the hand gesture was sensed and captured using a wrist-worn camera. In [33], the authors have used heart rate and skin conductance parameters for estimating the motivation and attention in due course of human-robot interaction. Agrigoroaie and Tapus have proposed a framework for behavior control that makes customized interaction between the robot and the patient with mild cognitive impairment. The models created will help the robot to interact with the patient both verbally and nonverbally [34]. In a recent study [35], the authors have reported the development of a socially assistive robot that enables people to maintain not only their health condition but also support them during social interaction. The designed robot can help the patients to improve their perception ability, social behavior, and provide structure for interaction. Furthermore, it can also change the feeling of a person [35]. Sharif and Alsibai have developed a “Nao Robot” that can analyze the medical data and interact with patients. After interaction with the robot, the patients will able to understand the vital signs of their body and make inferences regarding their health status [36]. Furthermore, it can predict the risk of heart diseases in the future and recommend the necessary changes in the lifestyle to avoid medical risks.

### 2.4. Cognitive Ability

The cognitive ability enables a robot to understand its relationship with the environment or a specific object. There are different aspects of cognition including perception, intelligence, encoding/decoding of information, reasoning, problem-solving, and thinking [37]. In an IoT-aided robotic environment, the robot makes use of the cloud and obtains knowledge from multiple sources, e.g., the human body and its surrounding environment. This helps the robot to create a virtual environment for simulating robot control policies. In IoT, cognitive techniques have been introduced recently in the management of distributed architecture. However, the inclusion of robots has not yet been sufficiently explored and demands more attention. In [38], the authors tried to design a cognitive architecture for the humanoid robot. The proposed architecture is the integration of a hierarchical module and a behavioral module. These modules were designed to keep the important aspects of cognition (e.g., perception, learning, planning, and motor control) in mind. This is to achieve a higher level of cognitive ability in the device. Literature suggests that cognition is interlinked with emotion and both are necessary to achieve a healthy social interaction [39]. This concept can be employed in the next-generation robotic systems for achieving a higher level of cognitive function.

### 2.5. Manipulation, Adaptation, and Decision-Making Ability

The basic application of a robot in an IoT environment is its ability to modify the sensor data [10]. In the healthcare environment, the robots can either be used for monitoring patient's health or detecting health abnormalities. In both cases, first, the robot has to acquire the health information using various sensors. This information follows various processing steps before providing meaningful information. The processing of the extracted data includes denoising, preprocessing, and thresholding. The implication of IoT technology in this process is to enable the integrated system to calculate those features that are not easily observable by the robots. Furthermore, a system needs to decide the best course of action to be taken during treatment. This can be achieved with help of a predictive algorithm designed using artificial intelligence, machine learning, or predictive analytics. However, the accuracy of predictions solely depends on the quality of the model and the efficiency in detecting the initial state. The integration of IoT provides a better perception and improves the decision-making ability of the integrated system. Again, it diversifies the ability of a robotic system in decision-making by integrating more sensors into the system. This will increase the information available to the predictive model and boost up the rate of accurate prediction. Another important functionality of the integrated system is its ability to work in a dynamic environment, which is called adaptability. This ability makes the system ready to deal with unforeseen events, faults, change in environmental conditions, tasks, or human behavior. Adaptability can be achieved with the help of other aforementioned abilities such as perception, cognitive, and decision-making. In [34], a robotic system was designed that can adapt and react based on the input user profile. Here, the profile information contains the level of disability, emotional states, personality, and preferences, etc. These robots can learn through their prior experience and adjust their behavior based on the individual response.

## 3. Application of IoT-Aided Robotic Technology in Healthcare

There are several fields in healthcare where the IoT and robotic technology have been efficiently employed in the past. Some of the most notable healthcare applications (Figure 3) of these technologies have been discussed. Furthermore, issues, challenges, and future implications are identified and reviewed in this section.

### 3.1. Rehabilitation

The employment of correct and scientific rehabilitative procedures plays an important role in the recovery of the motor ability of a patient [40]. The most common reason behind the motor disability may be a brain injury, chronic pain, stroke, tremor, etc. Among different rehabilitation categories, limb rehabilitation is the most common, which can be further classified into upper and lower limb rehabilitation. Rehabilitation training is difficult for many patients as it requires the help of a trained healthcare professional. An increase in cost, unavailability of medical staff, and geographical barriers make it difficult for these patients to access rehabilitative services. A more suitable solution for this problem is remote treatment using various home-based medical devices [41]. Over a decade, much-advanced technologies such as robotics, machine learning, and artificial intelligence have satisfied the need of many clinicians and patients in providing rehabilitation. A detailed description of the most commonly available technologies for limb rehabilitation is provided in [42, 43]. However, the application of IoT brings the patients, rehabilitative systems, and the physiotherapist into a common environment where they can work cooperatively. Numerous researches in the past have employed the IoT-aided robotic technology for rehabilitation [44–47]. Wai et al. have developed a low-cost portable home rehabilitation device that can improve various upper limb (hand, forearm, and wrist) movements. Li and Zhong have proposed an IoT-based upper limb rehabilitation system that was based on remote control [40]. Here, the pressure sensors are used as the source of control information. In [48], an IoT-aided robotic system for stroke rehabilitation has been reported that enables the doctors to remotely monitor the type, strength, and duration of the training at home. Furthermore, it will provide optimal prescription by analyzing the intensity of the rehabilitative training as feedback. Thakur et al. have used an accelerometer and a magnetometer sensor-based smart band that can recognize the hand motions such as flexion, extension, and adduction. The information collected from these sensors acts as a control signal for the robot that reflects the movement of the smart band [49]. In [50], an IoT-aided robotic system has been proposed that uses a natural user interface for rehabilitation. The system enables the therapists to record specific motions that will act as a control signal for the robot to create a similar motion in the patient's lower limb.

Despite the evolution of the aforesaid technologies, it is still a major challenge for the researcher to assemble the maximum skill of a physiotherapist. Although the IoT-aided robotic system is one of the most advanced tools, it is not a replacement for the physiotherapist. Presently, these systems are only capable of performing simple repetitive therapies. However, the importance of employing these technologies lies in the ability of a robot to provide longer and more intensive repetitive movements with the same consistency. The integration of IoT-technology enables physiotherapists to not only observe and manage multiple patients but also suggest the best suitable therapy for them. Moreover, it is important to give the patients a feeling of independence during their rehabilitation. This brings positivity and enhances their self-esteem. Hence, in future rehabilitation systems, the addition of various human movements is needed to design a multi-modal rehabilitation system. The ROBIN [51], a rehabilitative robot, was developed on a similar concept where the rehabilitation system not only provides stability to the trunk during a change in body position but also encourages the patients for simple arm and hand movements (reach and grasp). Current research in the said field is mostly exploring the use of augmented reality, videogames, and plays for rehabilitation. This is to increase the engagement and participation of the patients in the therapeutic process. It has also been reported that the use of video games during rehabilitative activities also improves motor function and hastens recovery. The cost of using a rehabilitation robot is still high as compared to drug-based or human-based therapies. This is limiting the wide-scale evaluation of these services and hence questioning their acceptance in the clinical practice. Also, a patient with restricted movement cannot pay regular visits to a hospital/rehabilitation center. Hence, in the future, efforts must be made for developing systems with low cost that will be suitable for an unsupervised environment. More attention is to be given to the adaptability of the rehabilitative systems so that they will work dynamically according to user needs. This may allow changing the therapeutic routine of the patients after evaluating the improvement in the patients' conditions.

### 3.2. Assistive Surgery

The invasive nature of the surgical procedure makes it a risky process. This provides a strong motivation for the use of numerous advanced state-of-the-art technologies to transform the conventional surgical process into minimally invasive and less complex. On that note, robotic technology is delivering a flexible work environment for surgeons and making the surgical process more precise and accurate. The use of the assistive robot requires continuous training for the surgeon and expertise in controlling the robotic system [52, 53]. Usually, the minimally invasive surgery is performed through a small incision point (diameter less than an inch) on the abdomen, which is also called the remote center of motion. Due to the use of a small incision point, controlling the robotic system involves multiple tasks such as control of surgical tip, handling the constraints generated at the incision point [54], and collision avoidance in the workspace [55]. The integration of the IoT technology enables the existing system to communicate and connect with external devices (such as wearable sensors, smart devices, and mobile phones), doctors, and nurses. An IoT-based surgical robot provides an environment where the surgeons can connect for teleoperation through the Internet. The advantage of using an IoT-aided robotic system is its increased operational workspace as compared to open surgery [56]. Numerous studies have been reported in the literature that have employed an IoT-aided robotic system in many applications including microsurgery, robotic assistive-minimally invasive surgery, and remote surgery [52, 57–59]. Ishak and Kit [60] have developed a robotic arm that can assist a doctor during surgery and take care of the patients. The robotic arm could be controlled through gesture and posture information. In [61], an IoT-based collaborative control scheme has been developed for robot-assistive minimally invasive surgery. The proposed scheme can handle multiple tasks on a priority basis and also ensure the control of motion constraints and collision during the surgery. Recently, the IoT-aided robotic system is also employing haptic technology [62] to enable the surgeon to operate the patients from an isolated part through the robotic interface [63]. Although the aforesaid field possesses the advantage of two widely used technologies, namely, IoT and Robotics, the major concerns of such systems include reliability, robustness, and security [64]. Furthermore, to make the system efficient and improve safety during surgery, it is essential to develop accurate models of both the human body and the robot characteristics. Proper validation of the systems developed for assistive surgery is also required before its commercialization. Despite the substantial growth, the employment of an IoT-aided robotic technology is still associated with few unique limitations that are making this field more challenging. Some of these limitations include establishing secure and adequate access, 2-D vision, restricted instrument flexibility, decreased depth perception, and reduced tactile feedback [65, 66]. Furthermore, the use of the Internet for the interconnectivity among various robots and the doctors may suffer from network disconnectivity, slow Internet speed, and service quality [57]. This may severely affect the accuracy and the success of a surgical procedure. The future of robotic surgery lies in developing more miniaturized devices, incorporating smarter instruments with the robotic system using IoT technology. These futuristic systems will be capable of sensing and informing the surgeon about various bodily parameters such as blood flow, tissue oxygenation, and tumor margin.

### 3.3. Prosthetics

According to the reports by the World Health Organization (WHO), more than 15% of the world's population is suffering from some form of disability [67]. If statistics are to be believed, 30 million people across the globe need an assistive device, out of which 10 million are amputees. Unfortunately, only 27–56% of the total upper-limb amputees and 49–95% of the total lower-limb amputees uses prosthetics [68]. Prosthetics are artificial body parts (limb, tooth, heart halve, and eye) that help a differently abled person to live independently with comfort. It not only compensates for the physical function but also the appearance of the lost part. The loss of a body part may be due to a tumor, accident, disease, trauma, or congenital defects. There is two common classification category for the prosthetic devices, i.e., either based on the way the prosthetic device receives power or the lost body part. Based on the received power source, it can be either body-powered or electrically powered. Various other sources of power, such as gas and hydraulics, have been proposed in recent years [69–71], but they lack in their practical applications. Similarly, based on the lost body part, the prosthetic can be classified into the limb, dental, somatic, and craniofacial prosthesis, among which the limb prosthetic is the most common and is further classified into the upper- and lower-limb prosthesis. The development of these prosthetic devices is time-consuming, complex, and involves a series of repetitive processes. This is due to the large variability in the size of the lost parts and also the response of the patient to these devices. In addition, the patient needs a thorough medical examination and training for the comfortable use of prosthetic devices. However, in recent years, prosthetic devices are becoming more realistic and comfortable for the patient with the application of more advanced technologies. Here, the contribution of robotic and IoT technologies in the development of various prosthetic devices has been discussed.

Lee et al. have developed a multi-fingered robotic hand that can mimic the hand movement more accurately [72]. The proposed robotic hand consists of four fingers on each hand and 12 joints that consist of linked knuckles and linear actuators. Under the project “Hand of Hope,” low-cost robotic hand prostheses with an efficient grasp control mechanism were developed that can perform object catch function [73]. In another study, a crude robotic hand has been proposed that resembles the human hand [74]. The hand was covered with a layer of artificial skin, which was made using soft silicon to give a feel and appearance of a real hand. It was capable of lifting small weights, up to 1.5 kg. The mechanism of the attachment used to create the movement of the body comes with its own disadvantage. Moving the prosthesis usually requires a large force. Furthermore, the number of control signals generated by the prosthesis is limited that restricts the movement with a lesser degree of freedom. A substitute to the body-powered control is the use of a myoelectric control mechanism where the electrical activity of the muscle contraction is used as a control mechanism. The myoelectric control works based on the basic principle of a “two-site two-state” [75]. Here, a pair of electrodes is placed on two different muscles where the contraction of one muscle causes opening while the other causes closing of the hand. Inspired by the working principle of the muscle-tendon system, Pfeifer et al. have developed a prosthetic hand (also called the Zurich-Tokyo hand) that gives a total of 13 degrees of freedom [76]. A high degree of freedom was achieved by tracking the joint movement using a set of sensors (tactile and nontactile). The sensors also measure the finger-space position. The advantage of a Zurich-Tokyo hand is: it can learn by itself while performing a movement or grasping an object. This was achieved by the morphology of the hand, the elastic tendons, and the deformable fingertips. However, the issue of the myoelectric control method is that finding two groups of muscles that give the opposite control is not always possible. The stochastic nature of the myoelectric signal results in error and inaccuracy of the system [77]. Also, the learning method involves the interpretation of the myoelectric signal by the user, which demands continuous training and mental efforts. Hence, other training modes and control mechanisms have been adopted for limb prosthetics [78, 79]. In a recent paper, an exoskeleton robot for the lower limb was developed that showed an efficient mass adjustment mechanism to maintain stability during movement. This helps the patients in correcting their posture [80].

Connecting the robotic prosthetic devices to the Internet and making them a part of IoT will enhance the device's productivity. The IoT technology enables the system to produce a rich information base for data processing. This helps in eliminating the issue of a lower degree of freedom as in the case of conventional limb prosthetics. Fukuda et al. have employed IoT technology to design a multifunctional prosthetic hand using a set of sensors placed on the objects, users, and the surrounding environment [81]. The collected information from these sensors is stored in the data management server. The control signal, generated after evaluating the collected information, is sent back to the prosthetic device. Moreover, the inclusion of smart sensors in the IoT-aided robotic environment provides an efficient feedback mechanism for the prosthetic system. In [82], the authors developed a mind-controlled robotic arm that is decorated with a smart sensor network. The smart sensors include a temperature sensor, pressure sensor, accelerometer, gyroscope, potentiometer, and proximity sensor. The electroencephalogram (EEG) signals were used for controlling the robotics arm whereas the set of smart sensors allowed the prosthetic device to interact with the surrounding environment. Li et al. have integrated IoT, artificial sensory perception, and haptic feedback to develop a robotic arm that can restore the grasping function in a patient [83]. Also, the system provides information at the point of contact that includes the surface properties and force of interaction. The integrated system improves the manipulation performance as well as the perception ability of the user.

In defiance of the improvement in the field of prostheses, there are still many issues that need to be addressed. One of the most basic challenges in designing a prosthesis is to achieve patient satisfaction. It has been reported that the desire for a prosthesis changes with time and with the individual. Also, there exists a complex relationship between a patient's desire for like-life replacement and the level of loss. For example, a patient with minimal loss wishes his prosthetic to be more natural, whereas a patient with a high level of loss prefers function more than appearance. This demands the customization of the prosthetic devices with human needs, loss, and cognitive ability [84, 85]. The control of a prosthetic device still needs high mental effort, which makes it inefficient for the patients having a mild cognitive disability. Though numerous studies have employed pattern recognition technology for controlling the prosthesis, the efficacy of this method is still unclear due to the lack of clinical evidence. Unfortunately, the cost of such devices is one of the major constraints in its popularization. The commercially available prosthetic devices range from $15000 to 100000 or even higher if additional customization is required [86]. Several research groups have worked for the development of low-cost prosthetic devices but they lack in their real-life application and catering to the customer need. This needs to be emphasized in the future.

### 3.4. Elderly Care

The population of elderly persons is growing rapidly. People above the age of 60 are expected to increase in number from 605 million (in 2000) to two billion (in 2050) [87]. Hence, there will be an increased need for a caregiver in the future. Although care centers and nursing homes provide services with other nutritional and social supports, they lack the feeling of independence. Elderly people usually prefer to live in their homes than living with residential care. This provides them a sense of individuality and comfort [88]. But, maintaining a healthy life at an older age without any support becomes difficult as aging is associated with various physical, sensory, and cognitive issues. Recently, the innovation in advanced technologies such as robotic technology, sensor technology, IoT, human-robot interaction, and navigation technology have provided potential solutions to the aforesaid issues by creating a physical environment for active aging [89]. The robotic system, which provides such an environment, is called a service robot. These service robots act as a companion for older people. Some of the most notable service robots reported in the past are Care-o-Bot, Aibo, CAESAR, JoHOBBIT, and PT2 [90, 91]. The service robot, with help of IoT technologies (sensors, RFID, GPS, infrared, and wearable sensors) connects the elderly with health professionals as well as family members. This helps them maintain a quality of life by providing reminders, fall detection, and interfacing with other home appliances.

In the last decade, several articles have reported the application of service robots in elderly care [92, 93]. Tanabe et al. have proposed a robot-operated elderly assistive system that combines the hand robot with an environmental control system [94]. In this case, the information assist system acts as a connecting link between the home automation and the remote location. Furthermore, with the integration of IoT, the system provides comfort and security. In [95], the authors proposed architecture for socio-technical development in elderly care. This is achieved by connecting both healthcare sensors and social robots into a common platform (Figure 4). The robotic system gives the physical health status of the elderly person by analyzing the various vital signs such as heart rate, temperature, and brain activities. The system also records the patient-reported outcome measure (PROMs) during their interaction with the robot. Combining the information from PROMs and the sensors, a health assessment report is generated at the end that will be available for the patient, caregivers, and doctors. One of the most common social challenges for the elderly population is mild cognitive impairment. A higher percentage of elderly people get affected with MCI. This leads to lower physical and cognitive performance in older people. Kostavelis et al. in their project “Robotic assistant for MCI patient at home (RAMCIP)” has designed a service robot that can efficiently support elderly people with MCI [96]. The designed system is capable of performing higher-level cognitive function through advanced human and environment perception mechanism that helps the robot to decide when to assist a patient. Fighting depression is another challenge for people who are living alone. Randall et al. have tested the feasibility of the socially assistive robot (SARs) as in-home therapeutic support for elderly persons who are dealing with depression [97]. The authors compared the human mental state of the elderly before and after the in-home installation of the robotic system. The results suggest that the assistive robot can be employed as a potential solution for in-home depression of the older population. The use of robotics in depression management for the elderly is also reported in [98–101]. Marques et al. have developed “AirBot” for the elderly to monitor indoor air quality using IoT technology [102]. Using the social network platform, the system alerts the caregiver when detecting poor air quality in the home environment. The system aims to improve the living environment for elderly people.

A major issue in the application of service robots in elderly care is their acceptance by professional caregivers. Although the recently developed assistive care systems are integrated with many advanced functions and features, they lack in their affordability. It is also essential to evaluate these systems based on their caregiving benefits. Moreover, the challenges they face during their practical implementations should also be considered for their acceptance by the elderly population. The second most important factor for the elderly population is their adaptation to advanced technology. Elderly people are slow learners and are not updated with the technology in comparison to the younger generation. This fact should not be avoided while designing the assistive system for the elderly. Most of these assistive systems work in a cooperative environment where the information is collected from various sensors and robots. This requires efficient data storage and management system.

### 3.5. Managing Disease Outbreak (COVID-19)

COVID-19, a novel respiratory syndrome disease, is now the most critical challenge to the world after the influenza pandemic outbreak of 1918 [103]. Many countries have been successful in reducing the spread of the infection, mortality, and morbidity associated with the disease. The cooperation of administration, healthcare system, and people played an important role in checking the spread of the disease. However, there are still some countries that are struggling to control the spread. This is due to the unpredictable nature of the virus in the human body. The new strain of the virus is the reason for its rapid outbreak. The virus is characterized by its highly contagious nature and the long incubation period (1–14 days). However, the recovery period may vary from 6 to 41 days depending on the person's age, health, and underlying conditions. The most common symptoms for the diagnosis of the disease include fever, cough, and fatigue, which are similar to flu symptoms. Also, it is possible that during this period, a person is infected but not showing any symptoms. In such cases, the infected person may act as silent carriers unknowingly; thus, making the disease highly contagious as compared to similar diseases in the coronavirus family. To alleviate the spread of the disease, various efforts with the use of advanced technologies have been suggested.

During the outbreak of a pandemic, the health workers are at a higher health risk. This is due to their direct contact with patients. The exposure of patients to health workers can be minimized if robots can be employed for some sort of nursing duty. Even though robotic technology has shown a wide range of healthcare applications (nursing, ambulance management, telemedicine, cleaning/disinfecting the hospital, reception, etc.), it failed to provide an effective solution in the fight against the pandemic. However, researchers have suggested various upgrades in healthcare robots that may help to deal with the COVID-19 pandemic (Figure 5). Nowadays, autonomous robots have been employed in the hospital premises to disinfect hospital wards, handle contaminated waste, and deliver medicine, food, or medical supplies to patients [104]. A wheeled telepresence robot can be employed in healthcare centers and hospitals for a virtual face-to-face patient assessment. The robots are capable of performing diagnostic tests after collecting the swab samples from the patients. This will facilitate the screening of patients while protecting the frontline health worker from direct contact. Indirectly, the robot reduces the time of exposure for health workers, avoids the use of personal protective equipment, and negates the chances of contamination during its removal. These robots can also be employed in crowded places such as airports, railway stations, and ports, where large-scale screening is necessary. Integrated with IoT technology, these robots can be used in various COVID-19-related applications. This includes checking whether a patient is following a quarantine rule or not, collecting temperature information from a remote location, and transmitting these data to healthcare centers to diagnose and alert patients about getting the COVID-19 infection. During quarantine, socially assistive robots may provide companionship to the patients and enable them to withstand social contact. For the elderly, and the physically impaired, the rehabilitation services can be continued with the help of robots without any physical contact with the therapist. In addition, mobile robots are installed in various public areas to check the maintenance of social distancing and the wearing of masks. Aerial robotics is used to supervise the quarantine areas and border control operations. In diagnosis, the teleoperated robotic system can play an efficient role in detecting the disease without the physical presence of the doctor. These systems can be used to check the pulmonary condition. In a recent study [105], a telerobotic system has been proposed for the cardiopulmonary assessment of the COVID-19 patients. Karmore et al. have developed a cost-effective medical diagnosis humanoid (MDH) that can provide a complete diagnostic test to check the COVID-19 infection [106]. In [107], the authors implemented an IoT-based drone technology to detect the coronavirus infection using the thermal images obtained from a thermal camera. Alsamhi and Lee have proposed a futuristic concept of collaborating multiple robots using blockchain technology and IoT to fight against COVID-19. This concept can be employed in the future for patient monitoring, outdoor, and hospital end-to-end delivery systems [108]. The technology is believed to manage multi-robot collaboration, improve interaction, and share health information more efficiently. In another study [109], the authors have developed a phone application infused with intelligent IoT features such as complex data analysis and intelligent data visualization for contact tracing of the infected persons. The intelligent data analysis techniques enable the system to improve public health and can be applied in the future health crisis.

In the future, IoT-aided robots may employ artificial intelligence and machine learning algorithms to detect the COVID-19 infection. A probable option can be the use of computer tomographic (CT) images for this purpose. The CT imaging technique has been used in many biomedical applications and is expected to be efficient in the diagnosis of COVID-19 infection. Some of the common biomedical applications of CT imaging include cancer detection [110], tumor identification [111], analysis of the interstitial lung images [112], pancreas segmentation [113], dental restoration, and tooth cavity detection [114, 115]. Recently, CT imaging is considered an effective method for the detection and monitoring of the symptoms of COVID-19 patients. These imaging methods have shown great potential in detecting the virus, especially in the case of asymptotic patients with negative nucleic acid testing [116]. Even though reliable criteria for the diagnosis of COVID-19 with CT-imaging technique have been developed (for example, the so-called effect of frosted glass), in practice, the volume of lung damage determined by CT does not always correspond to both the degree of lung damage and the severity of the development of pulmonary pneumonia. This also makes the development of IT methods for CT imaging highly relevant [107]. Herein, deep learnings can be applied for the analysis, interpretation, and tracking of a large number of CT data. While managing the COVID-19 infection, it is also crucial to look into the discharge criteria of a patient from the quarantine ward. The three most usual criteria include being nonfeverish for more than three days, resolved respiratory syndromes, improvement in the radiological signs for pulmonary illness, and a negative COVID-19 nucleic acid test. AI-based automated tools can be integrated with the IoT-aided robotic system to track the discharge criteria for patients with infection. In addition, it can be employed to differentiate healthy people from the infected ones.

## 4. Future Directions and Conclusions

The purpose of the current article was to give a comprehensive idea regarding the applicability of IoT and robotics technology in the current healthcare services. Furthermore, it provides a detailed description of the functionalities of an ideal IoT-aided robotic system for healthcare applications. Based on the above review, it is possible to say that although numerous studies have been dedicated to the healthcare applications of the aforementioned technologies, the field lacks controlled and clinical trials that will validate their practical applications. Whether it is the design of an assistive robot for surgery, a rehabilitative robot, a prosthetic device, or a smart-home for the elderly, the studies are mostly restricted to a future proposal or research projects. Hence, future studies must be highly focused on practical applications of these technologies and their acceptance in society. Furthermore, universal evaluation criteria must be employed for the developed devices. The evaluation should be followed by the implementation of various control strategies. This will help in maintaining the interconnectivity and interoperability of such devices, developed across the globe. A most common issue while employing these technologies in healthcare is measuring the success of the healthcare devices/systems and technology. This should be based on their ease of handling, cost, and satisfaction of patients and healthcare professionals. The real use of these technologies can only be assessed either by directly comparing them with the conventional methods or the way they are minimizing the efforts of the healthcare professionals. Various comparative studies on the same must be performed in the future. Also, the problems faced by the patients and healthcare professionals while operating these devices must be accessed and used as feedback for future development.

One of the drawbacks of the present robotic systems for healthcare applications is the limited scope for customization. The need for the customization of the healthcare service systems is of utmost importance for the healthcare professionals and patients, as the need varies from one patient to another. Hence, the current healthcare system demands more flexibility in the robot-based service devices that can easily adjust as per a patient's health status. The functioning of the robotic systems is highly influenced by the learning and training methodology used for their operation. Also, a prior study suggests that degradation of the skills has been observed in the case of newly trained robotic surgeons after a prolonged period of inactivity [117]. Hence, a new training methodology must be developed in the future, which not only enhances the device functionality but also its usability. For most of the studies, the cost is a major concern that restricts its wider application. A lower-cost system can significantly increase the popularity and acceptability of the system. Hence, more attention must be given to designing cheaper sensors and computer systems in the future. Furthermore, while installing a cooperative network as in the case of smart-homes, smart-hospitals, smart rehabilitative systems that integrate the IoT, various sensors, and robots, practical issues in their smooth functioning must be evaluated. This will enhance the acceptability and popularity of these systems in the future. Unfortunately, these systems have to deal with a large volume of information that is acquired from various sensors that are present in the network. The use of a high volume of data requires more advanced data management, analysis, and security techniques for the efficient use of the information. It has been reported that patients are adopting the newer technology but they are concerned about the privacy of their data. Hence, the patients must be aware and informed about the data sharing policies of the developed IoT-based robotic devices. Despite the claim of superiority of the IoT and robotic systems as compared to the traditional healthcare methods, these healthcare systems mostly depend on the skill and training of the patients and healthcare professionals for their efficient use. The aforementioned points will form a reference for future development in the said field. Also, the knowledge shared in the study will help the readers and future researchers to gain a comprehensive idea of the applications of the IoT-aided robotic technology in transforming healthcare services for people.

## Figures and Tables

**Figure 1:** A basic IoT-aided robotic healthcare system (modified from [14]).

**Figure 2:** Basic functionalities of an IoT-aided robotic system.

**Figure 3:** Some notable healthcare applications of IoT-aided robotic technology.

**Figure 4:** An ecosystem for elderly care that integrates healthcare sensors, robots, sensor networks, data processing unit, and a health assessment unit (reproduced from [95]).

**Figure 5:** Application of IoT-aided robotic system in managing COVID-19.

## Data Availability

No data were used to support this study.

## References

[1] Rong G., Mendez A., Bou Assi E., Zhao B., Sawan M. (2020). Artificial intelligence in healthcare: review and prediction case studies. *Engineering*.

[2] Belle A., Thiagarajan R., Soroushmehr S., Navidi F., Beard D. A., Najarian K. (2015). Big data analytics in healthcare. *BioMed Research International*.

[3] Ali O., Shrestha A., Soar J., Wamba S. F. (2018). Cloud computing-enabled healthcare opportunities, issues, and applications: a systematic review. *International Journal of Information Management*.

[4] Abdelaziz A., Elhoseny M., Salama A. S., Riad A. M. (2018). A machine learning model for improving healthcare services on cloud computing environment. *Measurement*.

[5] Gao J., Yang Y., Lin P., Park D. S. (2018). Computer vision in healthcare applications. *Journal of Healthcare Engineering*.

[6] Mehta N., Pandit A. (2018). Concurrence of big data analytics and healthcare: a systematic review. *International Journal of Medical Informatics*.

[7] Waring J., Lindvall C., Umeton R. (2020). Automated machine learning: review of the state-of-the-art and opportunities for healthcare. *Artificial Intelligence in Medicine*.

[8] Casola V., Castiglione A., Choo K.-K. R., Esposito C. (2016). Healthcare-related data in the cloud: challenges and opportunities. *IEEE Cloud Computing*.

[9] Patel A. R., Patel R. S., Singh N. M., Kazi F. S. (2017). Vitality of robotics in healthcare industry: an Internet of Things (IoT) perspective. *Internet of Things and Big Data Technologies for Next Generation Healthcare, Studies in Big Data*.

[10] Simoens P., Dragone M., Saffiotti A. (2018). The Internet of Robotic Things: a review of concept, added value and applications. *International Journal of Advanced Robotic Systems*.

[11] Akkaş M. A., Sokullu R., Çetin H. E. (2020). Healthcare and patient monitoring using IoT. *Internet of Things*.

[12] Postolache O., Hemanth D. J., Alexandre R., Gupta D., Geman O., Khanna A. (2020). Remote monitoring of physical rehabilitation of stroke patients using IoT and virtual reality. *IEEE Journal on Selected Areas in Communications*.

[13] Joseph A., Christian A., Abiodun A. A., Oyawale F. A. A review on humanoid robotics in healthcare.

[14] Rahmani A. M., Gia T. N., Negash B. (2018). Exploiting smart e-health gateways at the edge of healthcare internet-of-things: a fog computing approach. *Future Generation Computer Systems*.

[15] Afanasyev I., Mazzara M., Chakraborty S. Towards the internet of robotic things: analysis, architecture, components and challenges.

[16] Premebida C., Ambrus R., Marton Z.-C. (2018). Intelligent robotic perception systems. *Applications of Mobile Robots*.

[17] Hadidi R., Cao J., Woodward M., Ryoo M. S., Kim H., Letters A. (2018). Distributed perception by collaborative robots. *IEEE Robotics and Automation Letters*.

[18] Liu R., Chen T., Huang L. Research on human activity recognition based on active learning.

[19] Taylor R. H., Menciassi A., Fichtinger G., Fiorini P., Dario P. (2016). Medical robotics and computer-integrated surgery. *Springer Handbook of Robotics*.

[20] Fleming M., Patrick A., Gryskevicz M. (2018). Deployment of a touchless ultraviolet light robot for terminal room disinfection: the importance of audit and feedback. *American Journal of Infection Control*.

[21] Remy S. L., Blake M. B. (2011). Distributed service-oriented robotics. *IEEE Internet Computing*.

[22] Thrun S. (2007). Simultaneous localization and mapping. *Robotics and Cognitive Approaches to Spatial Mapping*.

[23] Khaliq A. A., Pecora F., Saffiotti A. Inexpensive, reliable and localization-free navigation using an RFID floor.

[24] Alotaibi M., Yamin M. Role of robots in healthcare management.

[25] Hou Y. C., Mohamed Sahari K. S., Yeng Weng L. (2020). Development of collision avoidance system for multiple autonomous mobile robots. *International Journal of Advanced Robotic Systems*.

[26] Fraga-Lamas P., Ramos L., Mondéjar-Guerra V., Fernández-Caramés T. M. (2019). A review on IoT deep learning UAV systems for autonomous obstacle detection and collision avoidance. *Remote Sensing*.

[27] Ahn H. S., Zhang S., Lee M. H., Lim J. Y., MacDonald B. A. Robotic healthcare service system to serve multiple patients with multiple robots.

[28] Safeea M., Neto P., Bearee R. (2019). On-line collision avoidance for collaborative robot manipulators by adjusting off-line generated paths: an industrial use case. *Robotics and Autonomous Systems*.

[29] Mišeikis J., Caroni P., Duchamp P. (2020). Lio-a personal robot assistant for human-robot interaction and care applications. *IEEE Robotics and Automation Letters*.

[30] Rodriguez-Losada D., Matia F., Jimenez A., Lacey G. Guido, the robotic SmartWalker for the frail visually impaired.

[31] Aly A., Tapus A. Towards enhancing human-robot relationship: customized robot’s behavior to human’s profile.

[32] Chen F., Lv H., Pang Z., Zhang J., Yang H., Yang G. (2018). WristCam: a wearable sensor for hand trajectory gesture recognition and intelligent human–robot interaction. *IEEE Sensors Journal*.

[33] Leite I., Henriques R., Martinho C., Paiva A. Sensors in the wild: exploring electrodermal activity in child-robot interaction.

[34] Agrigoroaie R. M., Tapus A. Developing a healthcare robot with personalized behaviors and social skills for the elderly.

[35] Chita-Tegmark M., Scheutz M. (2021). Assistive robots for the social management of health: a framework for robot design and human–robot interaction research. *International Journal of Social Robotics*.

[36] Sharif M. S., Alsibai M. H. Medical data analysis based on nao robot: an automated approach towards robotic real-time interaction with human body.

[37] Vanderelst D., Winfield A. (2018). An architecture for ethical robots inspired by the simulation theory of cognition. *Cognitive Systems Research*.

[38] Burghart C., Mikut R., Stiefelhagen R. A cognitive architecture for a humanoid robot: a first approach.

[39] Pessoa L. (2017). Do intelligent robots need emotion?. *Trends in Cognitive Sciences*.

[40] Li X., Zhong J. (2020). Upper limb rehabilitation robot system based on internet of things remote control. *IEEE Access*.

[41] Celesti A., Lay-Ekuakille A., Wan J. (2020). Information management in IoT cloud-based tele-rehabilitation as a service for smart cities: comparison of NoSQL approaches. *Measurement*.

[42] Jakob I., Kollreider A., Germanotta M. (2018). Robotic and sensor technology for upper limb rehabilitation. *PM&R*.

[43] Laferrier J. Z., Gailey R. (2010). Advances in lower-limb prosthetic technology. *Physical Medicine and Rehabilitation Clinics of North America*.

[44] Meng Q., Zhang H., Yu H. (2018). The Internet of Things-based rehabilitation equipment monitoring system. *IOP Conference Series: Materials Science and Engineering*.

[45] Naranjo-Hernández D., Talaminos-Barroso A., Reina-Tosina J. (2018). Smart vest for respiratory rate monitoring of COPD patients based on non-contact capacitive sensing. *Sensors*.

[46] Yao L., Sheng Q. Z., Benatallah B. (2018). WITS: an IoT-endowed computational framework for activity recognition in personalized smart homes. *Computing*.

[47] Balampanis S., Sotiriadis S., Petrakis E. G. M. (2016). Internet of things architecture for enhanced living environments. *IEEE Cloud Computing*.

[48] Meng Q., Zhang H., Yu H. An internet of things framework based on upper limb rehabilitation robots for rehabilitation.

[49] Thakur S., Das S., Bhaumik S. A smart-band operated wrist rehabilitation robot.

[50] Pavón-Pulido N., López-Riquelme J. A., Feliú-Batlle J. J. (2020). IoT architecture for smart control of an exoskeleton robot in rehabilitation by using a natural user interface based on gestures. *Journal of Medical Systems*.

[51] Loureiro R. C., Smith T. A. Design of the ROBIN system: whole-arm multi-model sensorimotor environment for the rehabilitation of brain injuries while sitting or standing.

[52] Su H., Sandoval J., Makhdoomi M., Ferrigno G., De Momi E. Safety-enhanced human-robot interaction control of redundant robot for teleoperated minimally invasive surgery.

[53] Su H., Yang C., Ferrigno G., De Momi E. (2019). Improved human-robot collaborative control of redundant robot for teleoperated minimally invasive surgery. *IEEE Robotics and Automation Letters*.

[54] Sandoval J., Su H., Vieyres P., Poisson G., Ferrigno G., De Momi E. (2018). Collaborative framework for robot-assisted minimally invasive surgery using a 7-DoF anthropomorphic robot. *Robotics and Autonomous Systems*.

[55] Zanchettin A. M., Ceriani N. M., Rocco P., Ding H., Matthias B. (2015). Safety in human-robot collaborative manufacturing environments: metrics and control. *IEEE Transactions on Automation Science and Engineering*.

[56] Okamura A. M., Simone C., O’leary M. D. (2004). Force modeling for needle insertion into soft tissue. *IEEE Transactions on Biomedical Engineering*.

[57] Guntur S. R., Gorrepati R. R., Dirisala V. R. (2019). Robotics in healthcare: an internet of medical robotic things (IoMRT) perspective. *Machine Learning in Bio-Signal Analysis and Diagnostic Imaging*.

[58] Akimana B.-T., Bonnaerens M., Van Wilder J., Vuylsteker B. (2016). A survey of human-robot interaction in the internet of things.

[59] Lehman A., Berg K., Dumpert J. (2008). Surgery with cooperative robots. *Computer Aided Surgery*.

[60] Ishak M. K., Kit N. M. Design and implementation of robot assisted surgery based on Internet of Things (IoT).

[61] Su H., Ertug Ovur S., Li Z. Internet of things (IoT)-based collaborative control of a redundant manipulator for teleoperated minimally invasive surgeries.

[62] Sreelakshmi M., Subash T. D. (2017). Haptic technology: a comprehensive review on its applications and future prospects. *Materials Today: Proceedings*.

[63] Kim S. S. Y., Dohler M., Dasgupta P. (2018). The internet of skills: use of fifth-generation telecommunications, haptics and artificial intelligence in robotic surgery. *BJU International*.

[64] Gatouillat A., Badr Y., Massot B., Sejdic E. (2018). Internet of medical things: a review of recent contributions dealing with cyber-physical systems in medicine. *IEEE Internet of Things Journal*.

[65] Baik S. H. (2010). *Robot Surgery*.

[66] Andrade A. O., Pereira A. A., Walter S. (2014). Bridging the gap between robotic technology and health care. *Biomedical Signal Processing and Control*.

[67] Casebolt M. T. (2020). Barriers to reproductive health services for women with disability in low-and middle-income countries: a review of the literature. *Sexual & Reproductive Healthcare*.

[68] Kumar P. K., Charan M., Kanagaraj S. (2017). Trends and challenges in lower limb prosthesis. *IEEE Potentials*.

[69] Bevilacqua V., Dotoli M., Foglia M. M., Acciani F., Tattoli G., Valori M. (2014). Artificial neural networks for feedback control of a human elbow hydraulic prosthesis. *Neurocomputing*.

[70] Schulz S., Pylatiuk C., Reischl M., Martin J., Mikut R., Bretthauer G. (2005). A hydraulically driven multifunctional prosthetic hand. *Robotica*.

[71] Peerdeman B., Boere D., Witteveen H. (2011). Myoelectric forearm prostheses: state of the art from a user-centered perspective. *Journal of Rehabilitation Research & Development*.

[72] Lee S., Noh S., Lee Y., Park J. H. Development of bio-mimetic robot hand using parallel mechanisms.

[73] Calderon C. A., Ramirez C., Barros V., Punin G. (2017). Design and deployment of grasp control system applied to robotic hand prosthesis. *IEEE Latin America Transactions*.

[74] Saikia A., Mazumdar S., Sahai N. (2016). Recent advancements in prosthetic hand technology. *Journal of Medical Engineering & Technology*.

[75] Scott R. N., Parker P. A. (1988). Myoelectric prostheses: state of the art. *Journal of Medical Engineering & Technology*.

[76] Pfeifer R., Iida F., Gomez G. (2006). Designing intelligent robots-on the implications of embodiment-. *Journal of the Robotics Society of Japan*.

[77] Hof A. L. (1991). Errors in frequency parameters of EMG power spectra. *IEEE Transactions on Biomedical Engineering*.

[78] Meng W., Liu Q., Zhou Z., Ai Q., Sheng B., Xie S. (2015). Recent development of mechanisms and control strategies for robot-assisted lower limb rehabilitation. *Mechatronics*.

[79] Farina D., Amsüss S. (2016). Reflections on the present and future of upper limb prostheses. *Expert Review of Medical Devices*.

[80] Huang G.-S., Chang S.-C., Chen C.-C., Lai C.-L. Development of lower limb exoskeleton robot.

[81] Fukuda O., Takahashi Y., Bu N., Okumura H., Arai K. (2017). Development of an IoT-based prosthetic control system. *Journal of Robotics and Mechatronics*.

[82] Beyrouthy T., Al Kork S. K., Korbane J. A., Abdulmonem A. EEG mind controlled smart prosthetic arm.

[83] Li G., Zhang L., Sun Y., Kong J. (2019). Towards the sEMG hand: internet of things sensors and haptic feedback application. *Multimedia Tools and Applications*.

[84] Biddiss E. A., Chau T. T. (2007). Upper limb prosthesis use and abandonment: a survey of the last 25 years. *Prosthetics & Orthotics International*.

[85] Mendez V., Iberite F., Shokur S., Micera S. (2020). Current solutions and future trends for robotic prosthetic hands. *Annual Review of Control, Robotics, and Autonomous Systems*.

[86] Kumar D. K., Jelfs B., Sui X., Arjunan S. P. (2019). Prosthetic hand control: a multidisciplinary review to identify strengths, shortcomings, and the future. *Biomedical Signal Processing and Control*.

[87] Gheorghiţă V. (2016). Anthropology and population: perspectives on aging. *Revista de Științe Politice. Revue des Sciences Politiques*.

[88] Secker J., Hill R., Villeneau L., Parkman S. (2003). Promoting independence: but promoting what and how?. *Ageing and Society*.

[89] Portugal D., Alvito P., Christodoulou E., Samaras G., Dias J. (2019). A study on the deployment of a service robot in an elderly care center. *International Journal of Social Robotics*.

[90] Do H. M., Pham M., Sheng W., Yang D., Liu M. (2018). RiSH: a robot-integrated smart home for elderly care. *Robotics and Autonomous Systems*.

[91] Pripfl J., Körtner T., Batko-Klein D. Results of a real world trial with a mobile social service robot for older adults.

[92] Abdi J., Al-Hindawi A., Ng T., Vizcaychipi M. P. (2018). Scoping review on the use of socially assistive robot technology in elderly care. *BMJ Open*.

[93] Vitanza A., D’Onofrio G., Ricciardi F., Sancarlo D., Greco A., Giuliani F. (2019). Assistive robots for the elderly: innovative tools to gather health relevant data. *Data Science for Healthcare*.

[94] Tanabe S., Saitoh E., Koyama S. (2019). Designing a robotic smart home for everyone, especially the elderly and people with disabilities. *Fujita Medical Journal*.

[95] Neef C., Richert A. (2020). Promoting autonomy in care: combining sensor technology and social robotics for health monitoring. *Engineering Proceedings*.

[96] Kostavelis I., Giakoumis D., Malasiotis S., Tzovaras D. RAMCIP: towards a robotic assistant to support elderly with mild cognitive impairments at home.

[97] Randall N., Bennett C. C., Šabanović S. (2019). More than just friends: in-home use and design recommendations for sensing socially assistive robots (SARs) by older adults with depression. *Paladyn, Journal of Behavioral Robotics*.

[98] Kargar B. A. H., Mahoor M. H. A pilot study on the eBear socially assistive robot: implication for interacting with elderly people with moderate depression.

[99] Randall N., Šabanović S., Chang W. Engaging older adults with depression as co-designers of assistive in-home robots.

[100] Moyle W., Cooke M., Beattie E. (2013). Exploring the effect of companion robots on emotional expression in older adults with dementia: a pilot randomized controlled trial. *Journal of Gerontological Nursing*.

[101] Šabanović S., Chang W.-L., Bennett C. C., Piatt J. A., Hakken D. A robot of my own: participatory design of socially assistive robots for independently living older adults diagnosed with depression.

[102] Marques G., Pires I. M., Miranda N., Pitarma R. (2019). Air quality monitoring using assistive robots for ambient assisted living and enhanced living environments through internet of things. *Electronics*.

[103] Nasajpour M., Pouriyeh S., Parizi R. M., Dorodchi M., Valero M., Arabnia H. R. (2020). Internet of Things for current COVID-19 and future pandemics: an exploratory study. *Journal of Healthcare Informatics Research*.

[104] Chamola V., Hassija V., Gupta V., Guizani M. (2020). A comprehensive review of the COVID-19 pandemic and the role of IoT, drones, AI, blockchain, and 5G in managing its impact. *IEEE Access*.

[105] Zhou H., Yang G., Lv H., Huang X., Yang H., Pang Z. (2019). IoT-enabled dual-arm motion capture and mapping for telerobotics in home care. *IEEE Journal of Biomedical and Health Informatics*.

[106] Karmore S., Bodhe R., Al-Turjman F., Kumar R. L., Pillai S. (2020). IoT based humanoid software for identification and diagnosis of Covid-19 suspects. *IEEE Sensors Journal*.

[107] Mohammed M., Hazairin N. A., Al-Zubaidi S., AK S., Mustapha S., Yusuf E. (2020). Toward a novel design for coronavirus detection and diagnosis system using IoT based drone technology. *International Journal of Psychosocial Rehabilitation*.

[108] Alsamhi S., Lee B. (2020). Blockchain for multi-robot collaboration to combat COVID-19 and future pandemics. http://arxiv.org/abs/2010.02137.

[109] Jahmunah V., Sudharshan V. K., Lih Oh S. (2021). Future IoT tools for COVID‐19 contact tracing and prediction: a review of the state‐of‐the‐science. *International Journal of Imaging Systems and Technology*.

[110] Farwell M. D., Pryma D. A., Mankoff D. A. (2014). PET/CT imaging in cancer: current applications and future directions. *Cancer*.

[111] Sun I.-C., Na J. H., Jeong S. Y. (2014). Biocompatible glycol chitosan-coated gold nanoparticles for tumor-targeting CT imaging. *Pharmaceutical Research*.

[112] Bartholmai B. J., Raghunath S., Karwoski R. A. (2013). Quantitative CT imaging of interstitial lung diseases. *Journal of Thoracic Imaging*.

[113] Roth H. R., Farag A., Lu L., Turkbey E. B., Summers R. M. (2015). Deep convolutional networks for pancreas segmentation in CT imaging. *Medical Imaging 2015: Image Processing*.

[114] Ausiello P., Ciaramella S., Garcia-Godoy F. (2017). The effects of cavity-margin-angles and bolus stiffness on the mechanical behavior of indirect resin composite class II restorations. *Dental Materials*.

[115] Solari D., Papallo I., Ugga L. (2020). Novel concepts and strategies in skull base reconstruction after endoscopic endonasal surgery. *Acta IMEKO*.

[116] Meng H., Xiong R., He R. (2020). CT imaging and clinical course of asymptomatic cases with COVID-19 pneumonia at admission in Wuhan, China. *Journal of Infection*.

[117] Sugihara T., Yasunaga H., Matsui H. (2018). A skill degradation in laparoscopic surgery after a long absence: assessment based on nephrectomy case. *Mini-Invasive Surgery*.

